The article "Overexpression of A613T and G462T variants of DNA polymerase β weakens chemotherapy sensitivity in esophageal cancer cell lines" was retracted in 2019. Reasons: duplicated images; unreliable data.

# Overexpression of A613T and G462T variants of DNA polymerase β weakens chemotherapy sensitivity in esophageal cancer cell lines

**DOI:** 10.1186/s12935-016-0362-x

**Published:** 2016-11-10

**Authors:** Yuanyuan Wang, Xiaonan Chen, Qianqian Sun, Wenqiao Zang, Min Li, Ziming Dong, Guoqiang Zhao

**Affiliations:** 1 School of Basic Medical Sciences, Zhengzhou University, No.100 Kexue Road, 450001 Zhengzhou, Henan China; 2 Collaborative Innovation Center of Cancer Chemoprevention of Henan, 450001 Zhengzhou, Henan China

**Keywords:** Esophageal cancer, DNA polymerase β, Mutation, Chemotherapy sensitivity

## Abstract

**Background:**

Human DNA polymerase β (polβ) is a small monomeric protein that is essential for short-patch base excision repair. It plays an important role in regulating the sensitivity of tumor cells to chemotherapy.

**Methods:**

We evaluated the mutation of polβ in a larger cohort of esophageal cancer (EC) patients by RT-PCR and sequencing analysis. The function of the mutation was evaluated by CCK-8, in vivo tumor growth, and flow cytometry assays.

**Results:**

There are 229 patients with the polβ mutation, 18 patients with A613T mutation, 12 patients with G462T mutation among 538 ECs. Analysis results of survival time showed that EC patients with A613T, G462T mutation had a shorter survival than the others (*P* < 0.05). CCK-8 and flow cytometry assays results showed the A613T, G462T EC9706 cells were less sensitive than WT cells to 5-FU and cisplatin (*P* < 0.05). Experiments results in vivo showed that the tumor sizes of A613T and G462T group were larger than WT and polβ^−/−^ groups (*P* < 0.05).

**Conclusions:**

In this study, we discovered A to T point mutation at nucleotide 613 (A613T) and G to T point mutation at nucleotide 462 (G462T) in the polβ gene through 538 EC patients cohort study. A613T and G462T variant of DNA polymerase β weaken chemotherapy sensitivity of esophageal cancer.

## Background

DNA polymerase β (polβ) is a protein which exists in mammalian cells [1]. Polβ belongs to the DNA polymerase family, and it is closely related to base excision repair (BER) [2–5]. BER is one of the most important DNA repair methods [6]. Through nonhomologous end joining, polβ participates in the repair of DNA double-strand break [7, 8].

Tumorigenes is involves a series of processes including genetic and epigenetic changes [9]. 30% of the tumors were reported to have a polβ mutation [10]. Abnormal expression of polβ leads to a highly mutagenic tolerance phenotype [11, 12]. Mutations polβ gene had been reported in a variety of cancers [13–17].

Esophageal cancer (EC) is one of the high incidence of malignant tumors in the world. Some research results showed that polβ gene mutation is exited in EC tissues [18, 19]. After lots of previous work, we discovered A to T point mutation at nucleotide 613 (A613T) and G to T point mutation at nucleotide 462 (A462T) in the polβ gene through 538 EC patients cohort study, and these two mutations are related to patients chemotherapy sensitivity. In this study, we analyze the relationship between polβ mutation and chemotherapy in ECs.

The article "Overexpression of A613T and G462T variants of DNA polymerase β weakens chemotherapy sensitivity in esophageal cancer cell lines" was retracted in 2019. Reasons: duplicated images; unreliable data.

## Methods

### Patients and tissue specimens

From 2000 to 2015, we collect a total of 538 tissues sample of EC patients in the First Affiliated Hospital of Zhengzhou University and Oncology Hospital of Linzhou City. The clinicopathologic characteristics of the 538 EC cases included in this study are presented in Table 1. Diagnosis by pathology experts, the tissues were stored in liquid nitrogen immediately. All patients were informed in advance and signed explicit informed consent. This study was approved by the ethics committee of Zhengzhou University.

**Table 1:** Clinicopathological characteristics of EC patients

Variables	Gender		Age		Tumor location		Lymph node metastasis		Differentiation			TNM stage		
	Male	Female	≥60	<60	Middle	Lower	Negative	Positive	Well	Moderate	Poor	I	II	III
n	365	173	337	201	421	117	323	215	151	269	118	154	263	121

### Cell and lentivirus infection of cells

EC cell line EC9706 and polβ null (polβ^−/−^) EC9706 cells [20] were established in our laboratory before. Full-length wild-type, A613T and G462T mutation polβ were amplified by PCR. These fragments were cloned into the lentiviral vector (LV5) to expression LV5-WT, LV5-A613T and LV5-G462T. Co-transfected 4.5 μg of that three LV5, 3.5 μg PG-P2-REV, 1.5 μg PG-P1-VSVG plasmids and 0.5 μg Lipofectamine2000 into 293T cells. Then we performed the lentiviral infection polβ^−/−^ EC9706 cells. When polβ^−/−^ EC9706 cells at a confluence of 60%, removed cell culture media. Culture cells with the virus-containing medium and polybrene. The MOI of lentiviral is 10. Stable cell lines were generated by puromycin selection. The cells were divided into four groups: wild-type EC9706 cells (WT), G462T mutation EC9706 cells (G462T), A613T mutation EC9706 cells (A613T) and polβ null EC9706 cells (polβ^−/−^).

### RNA isolation and RT-PCR

Using the Total RNA Kit I (R6834-01; Omega, USA) extracted RNA according to the manufacturer’s instructions. Then RNA was reversely transcribed to cDNA by reverse transcription Kit (Thermo, USA). The cDNA was performed PCR amplification. The fragments were extracted for agarose gel electrophoresis after PCR.

### DNA sequencing analysis

PCR amplification products were cloned into pGEM-T vectors, then transformed into DH5α *Escherichia coli.* Bacteria were amplified in liquid LB medium. The bacterial suspension was sent to sequencing analysis by Sangon Biotech (Shanghai).

The article "Overexpression of A613T and G462T variants of DNA polymerase β weakens chemotherapy sensitivity in esophageal cancer cell lines" was retracted in 2019. Reasons: duplicated images; unreliable data.

### qRT-PCR assay

With the extracted RNA, the first strand cDNA Synthesis Kit was used to synthesize cDNA with an oligo dT primer kit. TaqMan assays were used to detect the expression of polβ mRNA. Primers were designed by Primer Premier 5.0 software. PCR conditions were as follows: 50 °C 2 min; 95 °C 2 min; 95 °C 15 s, 55 °C 30 s, 72 °C 30 s, for 45 cycles. The 2^−ΔCt^ method was used to evaluate the relative expression of the target gene in the three groups. Primers sequences are as follows:

Forward: 5′ ACATGCTCACAGAACTCGCAAA 3′.
Reverse: 5′ TCCAGGCAATTTCTTAGCTTC 3′.
Probe: 5′ AAGAACGTGAGCCAAGCTATCCAC 3′.

We used β-actin as an endogenous control for normalization. Primers sequences are as follows:

Forward: 5′ AACCGCGAGAAGATGACCCA 3′.
Reverse: 5′ CACCGGAGTCCATCACGAT 3′.
Probe: 5′ CTGTGCTATCCCTGTACGCCTCT 3′.

### Western blotting

The total protein content of cultured cells was extracted using RIPA buffer containing phenylmethanesulfonylfluoride (PMSF). A BCA protein assay kit (Beyotime, Haimen, China) was used to determine the protein concentration. Proteins were subjected to sodium dodecyl sulfate polyacrylamide gel electrophoresis (SDS-PAGE) and transferred onto PVDF membranes. After blocking, the membranes were incubated overnight at 4 °C with diluted (1:300) primary antibodies (polyclonal rabbit anti-polβ; Proteintech). Following extensive washing, membranes were incubated with diluted (1:3000) horseradish peroxidase-conjugated goat anti-rabbit IgG (Santa Cruz). Signals were determined with a chemiluminescence detection kit (Amersham Pharmacia Biotech, Piscataway, NJ). An antibody against β-actin (Santa Cruz Biotechnology) served as an endogenous reference.

### CCK-8 assay

To confirm the effect of A613T and G462T mutation on chemotherapy, CCK-8 assay was performed in the four groups of EC9706 cells (WT, A613T, G462T, and polβ^−/−^). The drug concentration of 5-fluorouracil (5-FU) is 0–50 μg/mL, cisplatin is 0–8 μg/mL. The cells were seeded into a 96-well plate at a density of 3 × 10^4^/well. 24 h later removed the medium, washed by PBS for twice, and replaced with fresh medium drugs. After 48 h of drugs exposure, used Cell Counting Kit-8 (Dojindo, Kumamoto, Japan) to detect absorbance at 450 nm by Microplate Reader (Bio-Rad, Hercules, CA, USA). The experiment was repeated three times.

### Apoptosis assay

The four groups of EC9706 cells (WT, A613T, G462T and polβ^−/−^) were incubated overnight in complete medium. The attached cells were washed once with PBS, and then replaced with fresh medium containing 40 μg/mL 5-FU or 4 μg/mL cisplatin. Cells were harvested at 48 h post-transfection by trypsinization. Cells were resuspended at 10^6^ cells/mL in 1× binding buffer. After double staining with FITC-Annexin V and propidium iodide (PI) using the FITC Annexin V Apoptosis Detection Kit I (BestBio, Shanghai, China), cells were analyzed using an FACScan flow cytometer (BD Biosciences, USA) equipped with Cell Quest software (BD Biosciences).

The article "Overexpression of A613T and G462T variants of DNA polymerase β weakens chemotherapy sensitivity in esophageal cancer cell lines" was retracted in 2019. Reasons: duplicated images; unreliable data.

### *In vivo* tumor growth assay

Transfected with lentivirus of four groups cells (WT, A613T, G462T, and polβ^−/−^) (1 × 10^7^) were subcutaneously inoculated into 6-week-old female BALB/c nude mice at the dorsal flank. The mice were randomly divided into two groups: cisplatin group and 5-FU group. Each group had 5 mice. Cisplatin group was given to the mice in a dosage of 3 mg/kg, once weekly for 4 weeks. 5-FU was given to the mice in a dosage of 10 mg/kg, 2 days a time, and last 2 weeks. Then execute the mice to take out the tumor to survey tumor volume. All the operation of the mice is in line with the specification of National Institutes of Health.

### Statistical analysis

The software for statistical analysis is SPSS 21.0 (Chicago, IL, USA). Use *t* test and one-way analysis of variance to test difference among groups. Use the Kaplan–Meier and log-rank test to test the survival time. The difference was statistically significant when *P* < 0.05.

## Results

### A613T and G462Tmutations in esophageal cancer

In order to study polβ mutation in EC, we build a cohort of 538 EC patients. The mutations of polβ were detected by PCR and DNA sequencing. There are 229 (42.57%) patients with the polβ mutation (Table 2), 18 (3.35%) patients with A613T mutation, 12 (2.23%) patients with G462T mutation among 538 ECs (Fig. 1). A613T mutation takes in 7.86% of 229 polβ mutations, and G462T takes in 5.24% of 229 polβ mutations. The corresponding changes in amino acids of A613T and G462T mutations and their location in polβ protein are presented in Table 2.

**Table 2:** Mutations in 538 EC patients

Gene variation	n	Proportion %	Amino acid variation	Domain
375 nt: A → G	21	3.90	88 aa: I → V	8kD domain
454 nt: T → C	19	3.53	114 aa: F → S	Thumb domain
462 nt: G → T	12	2.23	117 aa: E → termination mutation	Thumb domain
466 nt: G → A	32	5.95	118 aa: G → E	Thumb domain
613 nt: A → T	18	3.35	167 aa: K → I	Palm domain
648 nt: G → C	20	3.72	179 aa: G → R	Palm domain
660 nt: A → G	27	5.02	183 aa: R → G	Palm domain
665 nt: T → C	8	1.49	184 aa: G → G	Palm domain
676 nt: G → A	15	2.79	188 aa: S → N	Palm domain
737 nt: A → T	6	1.12	208 aa: P → P	Palm domain
740 nt: A → G	9	1.67	209 aa: K → K	Palm domain
832 nt: A → G	11	2.04	240 aa: Q → R	Palm domain
853 nt: A → G	7	1.30	247 aa: E → G	Palm domain
854nt: A → C, and 855nt: A → C	12	2.23	247 aa: E → D, and 248 aa: K → Q	Palm domain
177–234 nt: deletion	12	2.23	22 aa: frameshift mutation; 26 aa: termination mutation	8kD domain
Total	229	42.57	–	–

GenBank Acc# M13140.1

The article "Overexpression of A613T and G462T variants of DNA polymerase β weakens chemotherapy sensitivity in esophageal cancer cell lines" was retracted in 2019. Reasons: duplicated images; unreliable data.

**Fig. 1:** DNA sequence analysis of ECs. Identification of the A613T and G462T mutations in ECs with DNA sequencing

### A613T and G462T mutations are related to the response to postoperative chemotherapy and shorten survival of EC patients

We analyzed the different survival time among patients with A613T, G462T mutation and others by Kaplan–Meier method. We used the Kaplan–Meier to analyze the difference in survival time between the patients with A613T mutation and wild type, the patients with A613T mutation and others (all patients except A613T mutation), the patients with A613T mutation and patients with other mutations (all patients with mutations except A613T mutation), based on follow-up visits of EC patients. The average survival time of patients with A613T mutation (18 cases) is 6.39 months, patients with wild-type (309 cases) is 38.35 months, and patients with other mutations (520 cases) is 30.89 months. Also, analyze the difference of G462T in the same way. The average survival time of patients with G462T mutation (12 cases) is 7.17 months, and patients with other mutations (526 cases) are 30.89 months. Analysis results show that EC patients with A613T or G462T mutation had a shorter survival than the others (*P* < 0.05, Fig. 2).

**Fig. 2:** Survival curves of ECs. **a**–**c** Patients with A613T mutation survival and the patients with wild-type polβ survival, others survival and other polβ mutation survival enrolled. **d**–**f** Patients with G462T mutation survival and the patients with wild-type polβ survival, others survival and other polβ mutation survival enrolled

### Polβ mRNA and protein expression levels in EC patients and cell lines

The expression levels of polβ mRNA and protein of patients samples and four groups cells (polβ^−/−^, WT, A613Tand G462T) were detected by qRT-PCR and western blot assays. Compared to adjacent non-tumor tissues, polβ mRNA expression in tumor tissue was found significantly higher (*P* < 0.05; Fig. 3a). All the EC patients’ samples were subjected to Western blot analysis, and the results were represented as polβ/β-actin. We randomly choose some samples as a representative. The polβ protein expression levels of adjacent non-tumor tissues of A613T mutation patients (A1–A3), G462T mutation patients (A4–A5), tumor tissues of A613T mutation patients (T1–T3, match to A1–A3) and polβ^−/−^, WT, A613T cell lines are presented in Fig. 3b. The standard error bars of patient samples are obtained from randomly selected patient samples, and the standard deviation bars of cell lines are obtained from three replications. The polβ protein expression levels of tumor tissues of G462T mutation patients (T4–T6, match to A4–A5) and G462T cell line are presented in Fig. 3c. We could find that the polβ protein expression levels of tumor tissues of these two mutation patients were significantly higher than that of adjacent non-tumor tissues (*P* < 0.05). There was almost no expression of polβ in the polβ^−/−^ cell line. polβ protein expression levels of WT, A613T, and G462T cell lines were significantly higher than that of adjacent non-tumor tissues (*P* < 0.05), and had no significant difference with tumor tissues.

The article "Overexpression of A613T and G462T variants of DNA polymerase β weakens chemotherapy sensitivity in esophageal cancer cell lines" was retracted in 2019. Reasons: duplicated images; unreliable data.

**Fig. 3:** Expression levels of polβ mRNA and protein of patients samples and four groups cells (polβ^−/−^, WT, A613T, and G462T). **a** Expression levels of polβ mRNA of patients samples. Compared to adjacent non-tumor tissues, polβ mRNA expression in tumor tissue was found significantly higher. **b** The polβ protein expression levels of adjacent non-tumor tissues of A613T mutation patients (A1–A3), G462T mutation patients (A4–A5), tumor tissues of A613T mutation patients (T1–T3) and polβ^−/−^, WT, A613T cell lines. **c** The polβ protein expression levels of tumor tissues of G462T mutation patients (T4–T6) and G462T cell line (*P < 0.05)

### A613T and G462T mutations weaken the proliferation inhibition effect of chemotherapeutics in EC9706 cells

In order to further study the relationship between polβ mutation and resistance to chemotherapy in ECs, we performed CCK-8 assay on four group cells for proliferation inhibition effect of 5-FU and cisplatin. The A613T, G462T cells were less sensitive than WT cells to 5-FU and cisplatin (*P* < 0.05; Fig. 4). The results were in agreement with the clinical observation, that A613T and G462T mutations patients have less chemotherapy sensitivity and short survival time, indicated that A613T, G462T mutation are associated with poor response to chemotherapy of ECs.

**Fig. 4:** Sensitivity of cell lines to cisplatin and 5-FU. **a** A613T and G462T mutations weaken the proliferation inhibition effect of 5-FU. Concentration of 5-FU was 0 to 50 μg/mL. **b** A613T and G462T mutations weaken the proliferation inhibition effect of cisplatin. Concentration of cisplatin was 0 to 8 μg/mL. WT: wild-type EC9706 cells; A613T: A613T mutation EC9706 cells; G462T: G462T mutation EC9706 cells; polβ^−/−^: polβ null EC9706 cells (*P < 0.05)

### A613T and G462T mutations weaken the apoptosis effect of chemotherapeutics in EC9706 cells

Our flow cytometry results indicated that the apoptosis levels of the A613T and G462T groups with 5-FU and cisplatin were weaken compared to the polβ^−/−^ and WT groups with5-FU and cisplatin (*P* < 0.05; Fig. 5). We conclude that A613T and G462T mutations weaken the apoptosis effect of chemotherapeutics in EC9706 cells.

The article "Overexpression of A613T and G462T variants of DNA polymerase β weakens chemotherapy sensitivity in esophageal cancer cell lines" was retracted in 2019. Reasons: duplicated images; unreliable data.

**Fig. 5:** A613T and G462T mutations weaken the apoptosis effect of chemotherapeutics in EC9706 cells. The apoptosis levels of the A613T and G462T groups with 5-FU and cisplatin were weaken compared to the polβ^−/−^ and WT groups with 5-FU and cisplatin (*P < 0.05)

### A613T and G462T mutations weaken the proliferation inhibition effect of chemotherapeutics in vivo

Experiments in vivo further confirmed the relationship between A613T, G462T mutation and poor response to chemotherapeutics. The tumor sizes of A613T and G462T group were larger than WT and polβ^−/−^ groups (*P* < 0.05; Fig. 6). These results indicated that A613T, G462T mutation weaken the inhibition proliferation of chemotherapeutics in vivo.

**Fig. 6:** The tumor volume of four groups. **a**,** b** The tumor tissues of four groups.** c**,** d** Tumor volume of four groups. Tumor volume of A613T and G462T groups were relatively bigger than WT and polβ-/- groups. polβ^−/−^: polβ null EC9706cells;WT: wild-type EC9706 cells; A613T: A613T mutation EC9706 cells;G462T: G462T mutation EC9706 cells. (*P < 0.05)

## Discussion

Esophageal carcinoma is one of the most common malignant tumors in the world. About 200,000 people die from esophageal cancer each year. There is great progress in the diagnosis and treatment of ECs, however, patients still have the problem of rapid progression and poor prognosis [21]. Surgery also has its disadvantages for patients and surgeons. The majority of EC patients with advanced choice of conservative treatment, such as chemotherapy. Chemotherapy is one of the main conservative treatments for EC. So far, the therapeutic efficiency of chemotherapeutics for EC has not been very well. The 5-year survival rate of EC wandered 10–30% and the probability of recurrence of the tumor is reached to 60–80% [22, 23]. Therefore, study of the factors that affect the sensitivity of chemotherapy is the focus of our research. In recent years, some genes have been reported that affect the sensitivity of chemotherapy, such as DNA damage repair proteins, apoptosis genes and cycle regulation genes [24–26].

Polymerase β closely related to BER for its polymerase and deoxyribose phosphate lyase activities. It also can maintain the integrity and stability of genomic [27]. polβ exists in a single nucleotide gap and leads to removal of the dRP group [28–30]. 30% of the tumors were reported to have a polβ mutation [10]. Many of these results are from a single amino acid substitution.

The article "Overexpression of A613T and G462T variants of DNA polymerase β weakens chemotherapy sensitivity in esophageal cancer cell lines" was retracted in 2019. Reasons: duplicated images; unreliable data.

The present study presents the A613T, G462T mutation of polβ gene in EC patients. The A613T, G462T mutations were associated with chemotherapy for EC. Some studies have shown that polβ exhibits opposite functions: an oncogene or as a tumor suppressor gene [31–33]. To detect the incidence of A613T, G462T mutation in EC, we established a cohort of 538 EC patients. The polβ mutation was detected in 229 (42.57%) of them. Among 229 polβ mutation cases, A613T point mutation was detected in 18 patients (7.86%) and G462T point mutation was detected in 12 patients (5.24%). The patients with A613T, G462T mutation had shorter survival time than the others. The results of CCK-8, flow cytometry and in vivo tumor growth assays indicated that polβ^−/−^ group cells are more sensitive than wild-type to 5-FU and cisplatin, and A613T, G462T mutation weaken the sensitivity of cells to 5-FU and cisplatin. The reason may be that polβ belongs to the DNA polymerase family, and it is closely related to BER, which is one of the most important DNA repair methods. That means polβ participates in the repair of DNA double-strand break. The A613T and G462T mutation may change some functions of polβ. Our clinical and experimental data indicate that A613T, G462T mutation has a tumor-promoting property, and in comparison to the wild-type polβ gene in EC, it may shorten survival of EC patients.

This study confirms that the A613T, G462T mutation of polβ desensitize EC patients to chemotherapy. Thus, the A613T, G462T mutation polβ gene may be clinically useful for EC patients to predicting the responsiveness to chemotherapy. It may serve as prognostic biomarkers for EC.

## Conclusions

In this study, we discovered A to T point mutation at nucleotide 613 (A613T) and G to T point mutation at nucleotide 462 (G462T) in the polβ gene through 538 EC patients cohort study. A613T and G462T variant of DNA polymerase β weaken chemotherapy sensitivity of esophageal cancer.

## Abbreviations

Polβ: DNA polymerase β
BER: base excision repair
EC: esophageal cancer
SDS-PAGE: sodium dodecyl sulfate polyacrylamide gel electrophoresis
PMSF: phenylmethanesulfonylfluoride
5-FU: 5-fluorouracil
PI: propidium iodide
